# Identification of Arrhythmia by Using a Decision Tree and Gated Network Fusion Model

**DOI:** 10.1155/2021/6665357

**Published:** 2021-05-29

**Authors:** Peng Lu, Yabin Zhang, Bing Zhou, Hongpo Zhang, Liwei Chen, Yusong Lin, Xiaobo Mao, Yang Gao, Hao Xi

**Affiliations:** ^1^School of Information Engineering, Zhengzhou University, Zhengzhou 450001, China; ^2^Collaborative Innovation Center of Internet Healthcare, Zhengzhou 450052, China; ^3^Department of Automation, School of Electrical Engineering, Zhengzhou University, Zhengzhou 450001, China; ^4^State Key Laboratory of Mathematical Engineering and Advanced Computing, Zhengzhou 450001, China; ^5^School of Software, Zhengzhou University, Zhengzhou 450002, China

## Abstract

In recent years, deep learning (DNN) based methods have made leapfrogging level breakthroughs in detecting cardiac arrhythmias as the cost effectiveness of arithmetic power, and data size has broken through the tipping point. However, the inability of these methods to provide a basis for modeling decisions limits clinicians' confidence on such methods. In this paper, a Gate Recurrent Unit (GRU) and decision tree fusion model, referred to as (T-GRU), was designed to explore the problem of arrhythmia recognition and to improve the credibility of deep learning methods. The fusion model multipathway processing time-frequency domain featured the introduction of decision tree probability analysis of frequency domain features, the regularization of GRU model parameters and weight control to improve the decision tree model output weights. The MIT-BIH arrhythmia database was used for validation. Results showed that the low-frequency band features dominated the model prediction. The fusion model had an accuracy of 98.31%, sensitivity of 96.85%, specificity of 98.81%, and precision of 96.73%, indicating its high reliability and clinical significance.

## 1. Introduction

Arrhythmia is a type of heart disease characterized by an irregular heartbeat with multiple categories and complex waveforms, making it difficult to accurately detect and locate waveforms and to set up classification features.

The traditional approach to arrhythmia identification is based on feature extraction (e.g., time-domain morphological features, frequency-domain features, and cardiac rhythm features) and the use of various machine learning classifiers, such as decision trees [1], nearest neighbor [2], support vector machines (SVMs) [3], logistic regression [4], and Artificial Neural Network [5]. These methods can often uncover potential explanatory factors hidden in observed sensory data, form abstract concepts, and reach consensus on recognition tasks [6]. However, feature design relies on the a priori knowledge of the designer.

In recent years, DNN technology has demonstrated excellent performance in the identification of cardiac arrhythmias. Several studies using recurrent neural network (RNN) variants of long short-term memory (LSTM) [7], convolutional neural network (CNN) [8], and other hybrid models have shown excellent performance in simplifying the input high-dimensional data into a compact low-dimensional representation space by automatically adjusting parameters using optimization algorithms. DNN creates end-to-end learning systems that use ECG signals as inputs and arrhythmia class predictions as outputs to automatically learn complex representative features from the data, reducing overreliance on artificially designed features. However, DNN, as an end-to-end black box model, has difficulty interpreting the significance of numerous parameters and the output of hidden neurons.

While the DNN black box approach may be sufficient in many use cases, models in sensitive medical areas need to provide a trustworthy basis for the validity of certain features on the identified results in order to understand the rationale behind the model's decisions and whether the decisions it makes are reliable. Improving the interpretability and reliability of the model is the core problem that needs to be addressed by clinically oriented algorithms for arrhythmia identification.

In this paper, a T-GRU fusion model is designed based on ECG time-frequency domain features and GRU networks. In this study, the gate recurrent unit (GRU) network model processes the time-domain features of the ECG signal, obtains the frequency-domain features of the ECG signal using the discrete FT, analyzes the discrete frequency-domain features through the decision tree, and finally weighs the fusion of the time-frequency domain feature output and gives the contribution of the time-frequency domain features of the fusion model to the results. The main areas of work in this study include the following:

1. Using the prior knowledge of the frequency domain and time domain of ECG data, the fusion algorithm is used to normalize the GRU model parameters and reduce the weight of its resultant output to improve the reliability of the fusion model
2. Decision tree probabilistic analysis of frequency domain features is introduced to discover the validity of low-frequency band features, and signal acquisition devices focusing on low-frequency bands can uncover more useful disease information
3. An incremental algorithm is designed to solve the problem of random selection of decision tree model band attribute nodes, and the algorithm improves the performance of the decision tree and fusion model

The remainder of the paper is organized as follows: Section 2 provides an overview of the T-GRU fusion model.  Section 3 presents the experiments and results.  Section 4 discusses the experimental results.  Section 5 concludes the study.

## 2. Related Work

Remote wearable monitoring devices enable continuous monitoring of cardiac activity, enabling better medical care for patients with cyclical dirty diseases. These devices record a large amount of raw electrocardiogram (ECG, electrocardiogram) data, which provides the data base for classification and identification using deep learning techniques.

Currently, deep learning techniques have achieved high recognition results for arrhythmia recognition identification. Several works use convolutional neural networks to detect abnormal ECG signals. Zubair et al. [9] introduced a convolutional neural network based ECG beat classification system. By using a small and patient-specific training data, the classification system effectively classifies ECG signals into five categories. Acharya et al. [10] developed a 9-layer deep convolutional neural network that can automatically identify five different types of heartbeats in ECG signals. Kiranyaz et al. [11] used a one-dimensional convolutional neural network for classification of ECG signals. Hannun et al. [12] developed a deep neural network which consists of 33 convolutional layers followed by a linear output layer to form a softmax.

A few works used recurrent neural network (RNN) models for the classification of heartbeats. Based on morphological information and temporal information, Wang et al. [13] applied a single RNN for automatic feature learning and classification. Zhang et al. [14] proposed a patient-specific ECG classification algorithm based on recurrent neural networks and density clustering techniques. Hochreiter et al. [15] proposed a long-time short-time memory (LSTM) recurrent neural network model that can effectively alleviate the long-distance dependence on RNNs.

However, deep learning methods map discrete category data for each domain into a representation suitable for neural network input, using deep information mining to automatically extract abstract features, and such abstract data features make it difficult for doctors to understand the basis for the model's classification.

But in reality, the model itself also implies knowledge, and doctors are more concerned with what the model learns from the data to produce decisions. If a model is completely uninterpretable, the application and deployment of the technology in the field of ECG identification will be limited by the inability to provide more reliable information.

Leveraging existing a priori knowledge of arrhythmias can improve model performance and the reliability of results. The local features of heartbeats are matrixed to generate global features [16], multilevel (beat, rhythm, and frequency level) domain knowledge features [17], and visual attention weights to improve model performance and interpretability. Gradient boosting trees are constructed to extract knowledge of cardiac behavior from DNNs to learn interpretable models and strong prediction rules [18]. The use of RNN to encode time variations in the 12-lead ECG signal sent to the attention module for advanced feature representation can be used for reliable diagnosis [19]. However, the main difference of this work is that the model has a high precision performance while providing a perceptually easy to understand contribution of frequency domain features from an energy point of view.

Deep learning-based ECG diagnostic algorithms can identify and determine arrhythmic events more effectively. However, deep learning techniques learn patterns and features of data from large amounts of data to represent output correlations rather than causal relationships. This causal uncertainty is key to the need for refinement of deep learning techniques, i.e., how to achieve effective classification recognition of ECGs, for reasons yet to be explored. To address the problem of arrhythmia recognition, it is necessary to explore a classification method that improves the credibility of deep learning models.

## 3. Materials and Method

### 3.1. Dataset

The MIT-BIH arrhythmia database is recognised as the definitive database of ECG heartbeat classification algorithms, and each record includes one-half hour segment of an ambulatory ECG with a 2-lead sampling rate of 360 Hz, for a total of approximately 650,000 sampling points. In total, there were over 109,000 marked beats from 15 different heartbeat categories, all marked by two or more cardiologists. In this paper, nonredundant 2-lead ECG signals are used to train and test our method.

### 3.2. Preprocessing

#### 3.2.1. Denoising

The discrete wavelet transform (DWT) [20] is used to denoise the original data. The WT is a time-frequency transformation method that analyzes the relationship between signals by varying the data on different scales. The usual discrete wavelet transform is:

(1) $$\begin{array}{c} \left(W_{\psi }f\right)\left(a,b\right)=<f,\psi_{a,b}>={\left|a_{0}\right|}^{-j2}\int_{-\infty }^{+\infty }f\left(x\right)\psi \bar{\left({a_{0}}^{-j}x-{nb}_{0}\right)}dt. \end{array}$$

Depending on the selection of the scale function, wavelet transforms at different scales can be obtained, with the scale transform being:

(2) $$\begin{array}{c} \varphi_{2^{j}}\left(x\right)=2^{j}\varphi \left(2^{j}\cdot x\right). \end{array}$$

The denoising results are shown in Figure 1, (a) the original signal and (b) the denoised signal.

As can be seen from the diagram, the method not only stops the noise from interfering but also effectively separates the signal from the noise.

#### 3.2.2. ECG Beat Segmentation

Excellent current R-peak detection algorithms have achieved over 99% positive predictability and sensitivity [21–28], and here, we have used the classical Pan-Tompkins algorithm to determine the R position, as in Figure 2. The R-peak reference point is taken as a heartbeat of about 0.3 s ahead and about 0.4 s behind, about 250 points. An example of a partial public heartbeat category after splitting is shown in Figure 3. (a) is normal beat, (b) is premature or ectopic supraventricular beat, (c) is ventricular escape beat, and (d) is fusion of ventricular and normal beat.

A specific classification developed by the Association for the Advancement of Medical Devices (AAMI) specifies that the 15 ECG waveforms in the MIT-BIH database can be classified into five categories: N (normal or bundle branch conduction block), S (supraventricular ectopic beats), V (ventricular ectopic beats), F (fusion beats), and Q (unassigned beats). Similarly to [29], the Q class was discarded because it has little representation in the database.  Table 1 shows the four categories of central beat data considered.

### 3.3. Frequency Domain Feature Extraction

The commonly used time-frequency domain conversion methods are FT, continuous wavelet transform (CWT), and Hilbert–Huang transform (HHT). Among them, HHT lacks strict physical meaning and mathematical support. Differences in the choice of CWT base functions may cause inconsistencies in the analysis results. The FT converts a time-domain signal into an easily analyzed frequency domain signal, i.e., a signal spectrum, which can be used to accurately calculate the composite modulus vector at each frequency. In addition, FT keeps the total amount of information constant during the transformation to the greatest extent possible.

The frequency domain feature segmentation depends on the QRS time-domain feature distribution interval. The QRS wave reflects the electrical behavior of the heart during ventricular contraction and has a large energy share. The discrete Fourier transform (DFT) was used to obtain the characteristics of each subband of the heartbeat. As in Figure 4, where (a) P-wave band, (b) QRS-wave band, and (c) T-wave band.

### 3.4. Methods

#### 3.4.1. Problem Description

The identification of arrhythmias can be translated into a multiclass task that can be structured using a softmax regression model as the last layer of the T-GRU (Figure 5) fusion model. The ECG time-domain training set *ℜ*_1_ is used as an input to the GRU model input layer and is output as the probability of each class of heartbeat. *ℜ*1 = {(*x*^(1)^, *y*^(1)^), ⋯, (*x*^(*i*)^, *y*^(*i*)^), ⋯(*x*^(*n*)^, *y*^(*n*)^)}, *x*^(*i*)^ is a time-domain signal sample, and *y*^(*i*)^ ∈ {0,1.2,3} is the class label of *x*^(*i*)^. The discrete Fourier transform is used to obtain the frequency domain training set *ℜ*_2_ as input to the decision tree and output as the corresponding label. Finally, the time-frequency domain output results are standardized and output through the fusion network model. Details are given in a subsequent section.

#### 3.4.2. GRU Model

GRU overcomes RNN's inability to handle long-range dependencies well, maintaining the effect of LSTM while making the structure simpler [30]. GRU is widely used in various time-domain scenarios, such as speech recognition and music and audio analysis [31], and is a good choice for ECG time-domain data classification.

As shown in Figure 6, the GRU model mainly consists of an input layer, a GRU network layer, and two fully connected layers. The input layer is the bottom component of the GRU model whose output is sent to the GRU network layer and is responsible for the preprocessing of the raw ECG time-domain data.

The GRU network layer consists of several GRU units (Figure 7) and is responsible for calculating the input hidden state as the first fully connected layer input. Each GRU unit consists of an update gate and a reset gate, with update gate *Z* deciding whether to update the new hidden layer state ${\tilde{h}}_{t}$ to the hidden layer state *h* and reset gate *r* deciding whether the previous hidden layer state is forgotten.

(3) $$\begin{array}{c} z_{t}=\sigma \left(W_{z}\cdot \left[h_{t-1},x_{t}\right]\right), \end{array}$$

(4) $$\begin{array}{c} r_{t}=\sigma \left(W_{r}\cdot \left[h_{t-1},x_{t}\right]\right), \end{array}$$

(5) $$\begin{array}{c} h_{t}=\tan h\left(w_{h}\cdot \left[r_{t}*h_{t-1},x_{t}\right]\right), \end{array}$$

(6) $$\begin{array}{c} {\tilde{h}}_{t}=\left(1-z_{t}\right)*{h_{t}}_{-1}+z_{t}*{\tilde{h}}_{t}. \end{array}$$

denotes two vectors connected, ∗ denotes the product of matrices, *σ* is the logical sigmoid function, tanh is the tangent function, and *x*_*t*_ is the input for the current *t* moment. *W*_*r*_, *W*_*z*_, and *W*_*h*_ are weight matrices that are learned during training and determined at the end of training.

The fully connected layer receives the hidden vectors from the network layer and outputs the classification results. Hidden vectors are learned on the last time step *h*_*t*_ and fed into the final classifier (softmax function) to perform the classification task. The classification task computes the probability that the predicted labels *y*_*k*_ in the *K* categories are *S*_*i*_.

(7) $$\begin{array}{c} S_{i}=\frac{e^{V_{i}}}{\sum_{i}^{k}e^{V_{i}}}. \end{array}$$

*i* represents the category index, *V*_*i*_ is the output of the classifier's previous output unit, and *S*_*i*_ represents the ratio of the index of the current element to the sum of all element indices.

#### 3.4.3. Incremental Decision Tree Model

The interpretative nature of tree classifiers is an important advantage over neural networks [32], which is suitable for capturing interactive information about discrete frequency domain features.

The decision tree model uses the CART algorithm. The “Gini index” is utilized to select the frequency complex mode vector attributes, and the Gini index classification for each leaf node in the tree is defined as follows:

(8) $$\begin{array}{c} \text{Gini index}=1-\underset{i}{\sum }{\left(\frac{n_{i}}{N}\right)}^{2}, \end{array}$$

where *N* represents the total number of frequency domain samples considered for that node and *n*_*i*_ represents the frequency domain signal label.

Pruning uses a cost-complexity-based approach with a loss function defined as follows:

(9) $$\begin{array}{c} C_{\alpha }\left(T\right)=C\left(T\right)+\alpha \left|T\right|. \end{array}$$

*T* is an arbitrary subtree, *C*(*T*) arbitrarily measures the fit of the training data, ∣*T*∣ measures the complexity of the tree, and *α* weighs the fit of the data against the complexity of the tree. *α* is taken from 0 to positive infinity to obtain the optimal subtree *T*(*α*) after pruning, and the output result is *D*_*i*_(1 ≤ *i* ≤ 4).

During the training of the decision tree, the criterion value of the frequency band attribute judgment is close to the critical value, and the node problem of splitting the random selection attribute occurs. Using an incremental algorithm (Algorithm 1), the decision tree training process eliminates junk samples to improve the generalization ability of the model, which is *ϑ*.

The sample data set was divided into ten equal parts, leaving 10% as the test set. For the remainder, an incremental algorithm was used, taking 10% of the samples at a time as the training set (9 times in total) and 80% as the validation set. The validation process is recorded as *Θ*. With constraint *f*, calculate the Gini index for all frequency attributes and then find the attribute with the largest Gini index to partition all data. This process is repeated for all partitions to obtain the spanning tree *T*_*k*_ to carry out the process *Θ* with *ϑ* and finally to generate the maximum subtree *T*_0_.

#### 3.4.4. Converged Network Model

As shown in Figure 8, the fusion network model is based on the CNN model with the aim of establishing a weight adaptive mechanism. The traditional approach to model fusion is linear weighting of fixed parameters, and in practice, the selection of parameters usually relies on lifting the global results. The CNN local sense field advantage facilitates learning local to global weighting information and adjusting the weighting dynamically. The CNN input is the weighting parameter *W*_*n*_^*i*^ after regularization of the GRU network model parameters.

The CNN network mainly consists of the weight input layer, Conv1D one-dimensional convolution layer, MaxPool1D one-dimensional pooling layer, GAPool1D global average one-dimensional pooling layer, dropout random inactivation layer, dense full connection layer, and softmax layer, where the first one-dimensional convolutional layer extracts the features of the weight *W*_*n*_^*i*^, the one-dimensional pooling layer convolutional kernel is 2 × 2, the step is 2, and the padding is “SAME.” Finally, the output of the CNN network is *W*_*i*_(1 ≤ *i* ≤ 2).

The goal of the fusion algorithm is to maximize the contribution of ECG frequency domain features to the weight of the fusion model results. The network weights of the GRU model are first attenuated using L2 regularization to reduce the overfitting of the model to some extent. The GRU model uses a cross-entropy loss function.

(10) $$\begin{array}{c} L_{i}=-s_{y_{i}}+\log\overset{k}{\underset{j=1}{\sum }}e^{s_{j}}. \end{array}$$

The linear scoring function corresponds to the correct category of *s*_*y*_*i*__.

(11) $$\begin{array}{c} C=L_{i}+\frac{\lambda }{2n}\underset{w}{\sum }w^{2}+0.001*W_{1}, \end{array}$$

where *L*_*i*_ represents GRU's cost function, (*λ*/2*n*)∑_*w*_*w*^2^ is the L2 regularization term, and *λ* is the regular term coefficient (0 < *λ* ≤ 0.1).

The output of the GRU model after L2 parameter regularization is softmax(∑_*n*_*W*_*i*_*h*). Moreover, the decision tree model output is *D*_*i*_.

The CNN network learning GRU global weights output *W*_*i*_. The decision tree model takes *W*_*i*_ with the largest weight as *W*_2_. Then, the GRU model weight is *W*_1_. Finally, the final result is output by the softmax function, and the fusion algorithm is as follows.

## 4. Experiments and Results

### 4.1. Experimental Data Division

In this paper, N, S, V, and F heartbeats were used as experimental data. The partitioned heartbeat data are randomly disordered. The ECG time-domain part is used as 80% as the training set, 10% as the validation set, and 10% as the test set. The frequency domain section is divided into ten equal portions of the sample data set, and the incremental algorithm is used.

### 4.2. Evaluation Indicators

The models were evaluated using sensitivity (Sen), specificity (Spe), precision (Pre), and accuracy (Acc). The formulas for calculating the four evaluation indicators are as follows:

(12) $$\begin{array}{c} \text{Sen}=\frac{\text{TP}}{\text{TP}+\text{FN}}, \end{array}$$

(13) $$\begin{array}{c} \text{Spe}=\frac{\text{TN}}{\text{TN}+\text{FP}}, \end{array}$$

(14) $$\begin{array}{c} \text{Pre}=\frac{\text{TP}}{\text{TP}+\text{FP}}, \end{array}$$

(15) $$\begin{array}{c} \text{Acc}=\frac{\text{TP}+\text{TN}}{\text{TP}+\text{FN}+\text{TN}+\text{FP}}, \end{array}$$

where TP (true positive) is the number of samples that predicted the abnormal signal as abnormal, TN (true negative) is the number of samples that predicted the normal signal as normal, FP (false positive) is the number of samples that predicted the normal signal as abnormal, and FN (false negative) is the number of samples that predicted the abnormal signal as normal. Acc indicates the overall classification accuracy of the overall model; Sen indicates the proportion of anomalous signals classified correctly, which measures the model's ability to identify anomalous signals; Spe indicates the proportion of normal signals classified correctly, which measures the classifier's ability to identify normal signals; and Pre indicates the proportion of signals classified as anomalous that are actually labeled as anomalous.

### 4.3. Experiment I

To verify the validity of the GRU model for time-domain signal detection, the segmented time-domain heartbeat sequence data were entered into the GRU network model (Figure 9).

After GRU network layer learning, the results were input to a fully connected softmax layer. To obtain better classification results, the network is constrained using the L2 regularization method. After 30 epochs, the GRU network converges, and the accuracy stabilizes as shown in Figure 9.

For cell effects, change the initial value of batch size and calculate the effect of different cells on the accuracy in 30 epochs.  Table 2 shows that the best accuracy is 97.52% when cell is 64.

For batch size effects, as shown in Table 3, the best accuracy obtained was 97.36 forbatch size = 128for an epoch of 30 and cell of 64.

Under optimal parameters, the Acc is 97.53%, the Sen is 95.3%, the Spe is 94.76%, and the Pre is 96.31%. The results show that the model is useful for automatic auxiliary analysis of ECG time-domain signals.

### 4.4. Experiment II

As in Figure 10, the effect of different frequency bands on the results of the decision tree model is verified without the frequency domain feature segmentation condition. The first five frequency bands are taken for the first time, and then, 20 additional frequency domain bands in sequence are used as input to the decision tree model. The DFT has conjugate symmetry, and the first 125 frequency bands are taken. Outputting their results as in Table 4, the accuracy of the first 45 bands differed from the first 125 bands by 0.13%, indicating that the lower band features were more important to the results.

To verify the performance of frequency domain data segmentation in the decision tree model, the classification results of frequency domain features without data segmentation are compared with those with data segmentation (Table 5). The results show that the data segmentation improves the performance of the model; the frequency domain data processing process is better interpreted by exploring each subwavelength using the decision tree model.

On the basis of frequency domain features with data segmentation, the training process uses an incremental algorithm.  Table 6 shows that the Acc is 96.68%, Sen is 95.03%, Spe is 94.43%, and Pre is 93.07%. The incremental algorithm further improves the performance of the model.

### 4.5. Experiment III

Under the incremental algorithm condition, the frequency domain data with segmented time-domain centroid sums are entered into the T-GRU fusion model. As shown in Table 7, the fusion model is significantly better than the single-domain, single-classifier model. And the sample weights *W*_2_ interval for CNN learning is for 0.59-0.68.

## 5. Discussion

In this paper, a T-GRU fusion model is designed to address the problem of identifying and diagnosing cardiac arrhythmias. The learning is based on ECG time-domain features and frequency domain features to improve the credibility of the deep learning model.

A decision tree with information entropy as a metric is introduced to analyze the contribution of each band feature to the prediction results using information expectancy. According to the standards published by the American College of Cardiology, the normal ECG signal frequency range is between 0.05 and 100 Hz, with 90% of the ECG spectral energy concentrated between 0.25 and 35 Hz [33]. As shown in Table 4, under the condition of no frequency domain data segmentation, the accuracy of the first 45 bands differs from the first 125 bands by 0.13%, which indicates that the decision tree model gives classification results mainly based on the low frequency bands, and the classification results have a certain degree of confidence. In addition, in practical applications, especially with signal acquisition equipment, the focus on the low frequency band when extracting features in the frequency domain can uncover more useful information about the disease.

QRS waves reflect the electrical behavior of the heart during ventricular contraction, with a large energy share, and are an important basis for the analysis of arrhythmias. The frequency domain characteristics of the individual subwaves are obtained based on the QRS waves, facilitating the analysis of information on the ECG signal loading of the individual subwaves. The experimental results are shown in Table 5. The frequency domain feature segmentation improves the classification performance of the decision tree model. The performance and credibility of the model is further improved by introducing some medical knowledge and using a decision tree model to explore the frequency domain data processing of each subwave.

The GRU network model uses deep information mining and automatically extracts abstract features of the ECG signal, which are difficult to understand due to the lack of causal relationship between such abstract features and the predicted results. To this end, a fusion network CNN is used to learn the weights of the time-domain data sample training and to assess the contribution of the data feature variables to the fusion results of the model. In Experiment 3, the sample weights *W*_2_ for CNN learning is 0.68, which indicates that under the regularized GRU network parameters, then the frequency domain features contribute more to the T-GRU fusion model results than the time-domain features, and the fusion model has some credibility.

The fusion model maintains a certain level of confidence while also taking into account the classification performance.  Table 8 gives the average evaluation results obtained using the T-GRU fusion model on the MIT-BIH dataset in comparison to other recent methods.

The T-GRU fusion model designed in this paper is, on average, just less accurate than Emina's method when the AAMI criteria are not used. Emina et al. used the discrete wavelet transform (DWT) to extract the wavelet coefficient features of the obtained frequency band representation distribution and finally used a random forest (RF) classifier in the diagnosis of ECG heartbeat signal classification. The AMMI standard specifies five main categories with a total of 15 different heartbeats. Emina's method of classifying arrhythmias was selected from only five; they are normal beat, left bundle branch block beat, right bundle branch block beat, atrial premature contraction beat, and premature ventricular contractions beat. This paper uses the AAMI criteria to actually select a total of 12 different heartbeats in four categories, N, S, V, and F. The average classification accuracy is just 1.02% lower.

The average accuracy of the method proposed in this paper is only 0.06% lower than WeiZhao's method when using the AAMI standard conditions. WeiZhao et al. Two leading heartbeat segments of length 2 s were generated on the filtered signal and classified by an adaptive ResNet model. The method has some advantages in terms of performance in classifying arrhythmias on ECG signals, and the lack of a basis for model decisions in an entirely DNN-based approach limits physicians' trust in such methods.

The fusion model provides a degree of confidence while maintaining high performance. However, frequency domain features have not yet been used extensively in clinical diagnosis, frequency domain features are less linked to medical knowledge, and a large amount of data is needed to determine their discriminatory criteria.

## 6. Conclusions

To address the problem of arrhythmia recognition, this paper focuses on exploring classification on methods to improve the credibility of deep learning models. A decision tree measured by information entropy as a metric is introduced to analyze the contribution of each frequency band feature to the prediction results. Fusion network CNN is used to assess the contribution of the data feature variables to the fusion results of the model. The experimental results show that the regularized GRU network parameters, particularly frequency domain features, contribute more to the results of the T-GRU fusion model than the time-domain features. The fusion model has a certain degree of credibility, which is of high reliability and clinical utility when applied to ECG automatic aid analysis.

Currently, frequency domain features are less associated with medical knowledge. To further enhance the trustworthiness of deep learning models, future research will explore medical linkage of frequency domain features or direct construction of trustworthy deep learning methods based on ECG time-domain features.

## Figures and Tables

**Figure 1:** Comparison of denoising results.

**Figure 2:** R-peak detection position.

**Figure 3:** Diagram of some types of heartbeat.

**Figure 4:** Example of subband segmentation.

**Figure 5:** Schematic of the fusion model. The leftmost part of the diagram is the GRU model dealing with time-domain sequences, the middle part is the CNN model of the fusion network learning GRU weights, and the rightmost part is the decision tree model dealing with frequency domain data.

**Figure 6:** GRU model.

**Figure 7:** GRU unit structure.

**Figure 8:** Convergence network CNN.

**Figure 9:** GRU training result chart: (a) training loss value; (b) overall Acc and individual Acc values.

**Figure 10:** Global characterization of the frequency domain.

**Algorithm 1:** Incremental algorithm.

**Algorithm 2:** Fusion algorithm.

**Table 1:** Five types of heartbeat data.

	MIT database heartbeat comment information		Total
AAMI provision of the heartbeat category	N	Normal beat	90081
		Left bundle branch block beat	
		Right bundle branch block beat	
		Nodal (junctional) escape beat	
		Atrial escape beat	
	S	Aberrated atrial premature beat	2781
		Nodal (junctional) premature beat	
		Atrial premature beat	
		Premature or ectopic supraventricular beat	
	V	Premature ventricular contraction	7008
		Ventricular escape beat	
	F	Fusion of ventricular and normal beat	802
	Q	Paced beat	72
		Unclassifiable beat	
		Fusion of paced and normal beat	

**Table 2:** Classification accuracy of different cell.

Cell	8	16	32	64	128	256
Acc (%)	96.13	96.56	97.21	97.52	97.31	97.26

**Table 3:** Classification accuracy of different batch sizes.

Batch_size	16	32	64	128	256
Acc (%)	83.1	85.21	94.32	97.36	92.23

**Table 4:** Classification performance evaluation of different frequency bands.

Frequency band	Sen (%)	Spe (%)	Pre (%)	Acc (%)
5	81.23	76.02	85.37	92.23
25	90.11	82.73	89.61	95.19
45	93.23	91.02	91.17	95.21
65	93.03	91.46	91.35	95.25
85	93.47	91.77	91.37	95.26
105	93.61	91.75	91.42	95.31
125	93.63	92.15	91.59	95.34

**Table 5:** Influence of frequency domain feature segmentation on classification performance.

Segmentation	Sen (%)	Spe (%)	Pre (%)	Acc (%)
With	93.68	92.23	91.65	95.41
Without	93.59	92.17	91.60	95.32

**Table 6:** The effect of incremental algorithm on classification performance.

Algorithm	Sen (%)	Spe (%)	Pre (%)	Acc (%)
Incremental	95.03	94.43	93.07	96.68
Without incremental	93.67	92.19	91.71	95.43

**Table 7:** Overall classification performance.

Algorithm	Sen (%)	Spe (%)	Pre (%)	Acc (%)
Tree	95.07	94.46	93.05	96.67
GRU	95.9	94.72	96.33	97.52
T-GRU	96.85	98.81	96.73	98.31

**Table 8:** Comparison of related work.

Works	AAMI	Classes	Methods	Acc	Sen	Pre
Zhao et al. [34]	Yes	4	ResNet	98.37	97.68	93.01
Liu et al. [35]	Yes	4	CNN + LRSVM	95.63	68.72	81.46
Zhou et al. [36]	Yes	5	LSTM	98.02	90.14	88.03
Shan et al. [37]	No	5	2D-CNN	97.56	95.97	95.61
Gad et al. [38]	No	2	DSNT + SVM	92.16	51.93	59.53
Li et al. [39]	Yes	5	WPE + RF	95.63	78.79	91.51
Emina et al. [40]	No	4	DWT + RF	99.33	**—**	**—**
Sena et al. [41]	No	3	CNN	97.75	95.42	94.3
Qin et al. [42]	No	6	WMRA + SVM	94.64	62.81	77.41
Amna et al. [43]	Yes	3	ESBMM + CNN	93.58	—	—
Our work	Yes	4	T-GRU	98.31	96.85	96.73

## Data Availability

The data used to support the findings of this study are included in the article. Further data can be requested from the corresponding author.
